The article "Ultrasound-Guided Stellate Ganglion Block Combined with Extracorporeal Shock Wave Therapy on Postherpetic Neuralgia" was published in 2022. Journal: J Healthc Eng.

# Ultrasound-Guided Stellate Ganglion Block Combined with Extracorporeal Shock Wave Therapy on Postherpetic Neuralgia

**DOI:** 10.1155/2022/9808994

**Published:** 2022-01-07

**Authors:** Changsheng Wang, Fei Yuan, Lu Cai, Haiqin Lu, Gongjin Chen, Jinping Zhou

**Affiliations:** Department of Anesthesiology, Shaoxing Second Hospital, Shaoxing 312000, Zhejiang, China

## Abstract

**Objectives:**

To evaluate the effect of ultrasound-guided stellate ganglion block combined with extracorporeal shock wave therapy (ESWT) on postherpetic neuralgia.

**Methods:**

Thirty-six patients with craniofacial postherpetic neuralgia, whose skin lesions were healed and natural course more than 1 month, were selected for the study and then randomly divided into 3 groups: the ultrasound-guided stellate ganglion block group (group A, *n* = 12), the extracorporeal shock wave therapy group (group B, *n* = 12), and the combined treatment group (group C, *n* = 12). Each group received basic drug treatment. The Visual Analogue Scale (VAS) and the Pain Disability Index (PDI) were used to evaluate the clinical effects of the 3 groups of patients before treatment, after twice treatments, after treatment for four times, and after treatment for six times.

**Results:**

The VAS and PDI were significantly declined in each group after the treatment (*P* < 0.05), and the declination in group C was more obvious than the other two groups (*P* < 0.05). After treatment for six times, the VAS score of group A, group B, and group C was 3.1 ± 1.2, 3.3 ± 1.3, and 1.9 ± 0.7, respectively. After treatment for six times, the PDI of group A, group B, and group C was 11.7 ± 8.4, 12.3 ± 7.8, and 4.6 ± 3.2, respectively. Three patients developed skin bruising and slight swelling, which were relieved by themselves.

**Conclusions:**

Ultrasound-guided stellate ganglion block combined with shock wave therapy could significantly improve the pain symptoms of patients with postherpetic neuralgia, which is a safe and effective treatment for postherpetic neuralgia.

## 1. Introduction

Postherpetic neuralgia (PHN) is a common clinical neuropathic pain. It is a pain that lasts for 1 month or more after healing of the herpes zoster (HZ) rash [1] and is the most common complication of herpes zoster. According to statistics, the total incidence of neuralgia after acute herpes virus infection is 9–34%, and the incidence is as high as 65–73% in patients over 60 years old [2]. The pain is severe and is a refractory disease, mostly manifested as spontaneous pain, hyperalgesia, abnormal pain, and paresthesia, causing patients to sleep and eat, emotional restlessness, and seriously affecting the quality of life and normal work. Therefore, timely and effective control of pain and improvement of patients' quality of life have become the focus of rehabilitation of patients with postherpetic neuralgia.

At present, drug treatment, nerve block, and radiofrequency therapy are often recommended in the treatment guidelines for PHN, but only 40–50% of patients have achieved satisfactory efficacy [3]. The mechanism of stellate ganglion block (SGB) in the treatment of pain is to improve the blood supply of the head and neck, inhibit the overexcitement of sympathetic nerves, regulate endocrine system, and relieve pain; at the same time, it can reduce the patients' fear, anxiety, and other symptoms and improve immune function, and enhance anti-inflammatory effect [4]. As a noninvasive method, extracorporeal shock wave therapy (ESWT) can generate tensile and compressive stresses through shock waves, causing piezoelectric effects and cavitation effects, changing the cell potential of local lesions, generating charge change, and exerting biological effects. It also produces physical effects in the soft tissues to release adhesions and relieve pain [5].

At present, the treatment of postherpetic neuralgia is mostly comprehensive treatment, but there is no report on the combined treatment of SGB and ESWT for PHN, and there are few reports on the impact on the quality of life. In this study, the combined application of SGB and ESWT was used to give full play to each other's advantages in the treatment of PNH and compared with a single treatment to comprehensively evaluate the clinical efficacy and safety.

## 2. Materials and Methods

### 2.1. General Information

From January 2018 to June 2020, 36 patients who were diagnosed with postherpetic neuralgia (the pain areas are mainly chest, head, and face) and met the inclusion criteria were selected in the pain clinic of our hospital. Among them, 20 were males and 16 were females, aged 52–88 years old, with an average of 69.8 ± 9.7 years old. There was no statistically significant difference in general information such as age, gender, and disease course of the patients (*P* > 0.05). This study was approved by the ethics committee of our hospital, and each patient signed an informed consent form before enrolling the cases.

*Inclusion Criteria.* (1) According to the patient's medical history, physical signs, clinical symptoms, physical examination and auxiliary examination, the patient was clearly diagnosed as PHN by a clinically experienced pain physician. (2) The skin lesions have healed. (3)Severe, persistent, stubborn pain, local skin numbness, hyperalgesia, and paresthesia. (4) The course of the disease is more than 1 month.

*Exclusion Criteria.* (1) Patients with severe allergies to related drugs. (2) Patients with bleeding tendency diseases and abnormal blood coagulation. (3) Infections in relevant parts of the treatment. (4) Patients with heart, lung, liver, kidney, and other important organic diseases. (5) Patients with cognitive impairment or mental illness. (6) Patients who cannot make a definitive and effective evaluation of the therapeutic effect of this study. (7) Patients with nausea, vomiting, dizziness, urinary retention, and other conditions before enrollment.

### 2.2. Research Methods

Three groups of patients were given basic drug treatment: gabapentin capsules (Jiangsu Enhua Pharmaceutical Co., Ltd.); the initial dose was 300 mg per day and slowly titrated to the effective dose. The usual effective dose was 900–3600 mg per day [6].

Group A: ultrasound-guided stellate ganglion block treatment. Select the PHN ipsilateral stellate ganglion for block therapy, in the horizontal paratracheal approach of the sixth cervical vertebra; the patient was in supine position; the ultrasound was conducted with a linear probe (10 MHz); and the probe direction was about 30° angle with the sagittal position of the neck. The needle can be inserted in the ultrasound plane, reached the surface of the longus cervicalis, no blood was drawn back, and 0.2% ropivacaine 5 ml was injected. The patient presented with Hornor syndrome: blocked lateral enophthalmic entrapment, dilated pupils, ptosis, increased skin temperature of the head, face and limbs, and decreased sweat gland secretion in the face and neck and other signs. The block was successful. After the treatment is completed, bed rest was required in the consulting room for 30 minutes. Once a week, 6 times is a course of treatment.

Group B: the MP100 shock wave therapy system of German STROZ company was used for treatment. The pain feedback method was used to locate the treatment area. The percussive pain point was first touched and marked, the coupling agent was applied, and the shockwave treatment was conducted along the ganglia with the tenderness point as the center; each impact is 4000–6000 times, frequency is 8–12 Hz, and pressure is 100–300 kPa. The corresponding probes were selected according to different treatment sites. The initial energy was the frequency of 8 Hz, and pressure was 100 kPa. The energy output was increased or decreased as appropriate according to the pain score and tolerance of the patients' feedback. The VAS score is controlled at 7-8 points. Important nerve trunks, large blood vessels, and lungs were avoided during treatment. The treatment was generally carried out in the outpatient clinic. After the treatment, the patients were told to drink more boiled water to promote metabolism. If discomfort such as redness, ecchymosis, and other discomfort occurs after the operation, apply a cold compress and wait for it to subside naturally. Once a week, 6 times is a course of treatment.

Group C: combined two treatment plans, once a week, 6 times as a course of treatment.

### 2.3. Judgment of Curative Effect

The visual analogue scale (VAS) was used to judge the degree of pain. Draw a 10-centimeter horizontal line on the paper; one end of the horizontal line is 0, indicating no pain; the other end is 10, indicating unbearable pain; the middle part indicates different degrees of pain. The patient draws a mark on the horizontal line according to self-feeling to indicate the degree of pain. Scoring criteria: 0 points, no pain symptoms; 1 to 3 points, mild pain, do not affect daily activities; 4 to 6 points, moderate pain, affecting daily rest during attacks; 7 to 10 points, severe pain, must stay in bed when the attack.

Quality of life (QOL) score, using Pain Disability Index (PDI) [7] to self-test the impact of chronic pain caused by PHN on patients' daily life, including family/family responsibilities, entertainment, social activities, work, sexual behavior, life support behavior, and other 7 items; each item is 0–10 points, 0 points means no impact, 10 points means that the behavior is interrupted or prevented by pain and cannot be performed at all. The total score is 70, and the lowest is 0. The higher the score is, the more obvious the impact on the quality of life is.

### 2.4. Statistical Analysis

Statistical analysis was performed using SPSS 25.0 software. Measurement data were expressed in the form of mean ± standard deviation (*x* ± *s*), one-way ANOVA was used for comparison between groups, LSD-T test was used for further comparison between the two groups, and *χ*^2^ test was used for counting data. *P* < 0.05 indicates that the difference is statistically significant.

## 3. Results

### 3.1. VAS Score

VAS in all three groups decreased after treatment compared with before treatment, the difference was statistically significant (*P* < 0.05). VAS decreased more significantly in the combined treatment group (group C) (*P* < 0.05). Results were showed in Table 1.

### 3.2. NPS Score

After treatment and before treatment, the PDI of the three groups decreased, and the difference was statistically significant (*P* < 0.05). On comparison between the groups, the PDI of the combined treatment group (group C) was more significantly decreased (*P* < 0.05) as shown in Table 2.

### 3.3. Safety Evaluation

Neither group A nor group C had nerve block-related complications and adverse reactions. A total of 3 patients in groups B and C showed skin bruises and slight swelling, and the symptoms resolved spontaneously after rest, and no other complications occurred.

## 4. Discussion

Postherpetic neuralgia is the most common and most serious complication of herpes zoster, and it is a chronic neuropathic pain. In recent years, the total incidence of PHN has been increasing, and the incidence and prevalence of herpes zoster and PHN has gradually increased with age. With the development trend of aging population in modern society, the number of PHN patients will further increase in the future. In recent years, scholars at home and abroad have conducted a lot of research on PHN, but its mechanism is still not completely clear. The current guidelines believe that neuroplasticity is the basis of PHN generation, and its mechanism [8] may include peripheral and central sensitization and a series of pathophysiological changes such as abnormal increase in the excitability of related neurons or enhanced synaptic transmission that cause the pain threshold to decrease and pain signal amplification. The corresponding clinical manifestations mainly include spontaneous pain, allodynia, and hyperalgesia in the affected area. PHN manifests as severe and intractable pain, often electric shock-like, burning-like, tear-like or knife-cutting pain, and it is also often accompanied by hyperalgesia, night pain, and paresthesia. 30–50% of patients have a disease course of more than 1 year, and some patients' pain lasts for more than 10 years [9]. Long-term pain causes moderate to severe disturbances in emotions, sleep, and life of patients, which seriously affects the quality of life and daily work of patients. At present, drug treatment for PHN is more complicated and has many adverse reactions. Therefore, it is particularly important for PHN patients to adopt reasonable treatment methods to effectively control pain as soon as possible, reduce drug dosage and adverse reactions, improve sleep and emotional disorders, and improve the quality of life.

Ultrasound-guided stellate ganglion block is a minimally invasive treatment method. Its main effect is divided into two aspects: central and peripheral. The central effect is mainly in the hypothalamus. It has the function of regulating the autonomic nervous system, endocrine system, and immune system and helps maintain the stability of the body's environment and normal cardiovascular function [10]. Its peripheral function is to inhibit sympathetic nerve innervation vasoconstriction, glandular secretion, muscle movement, bronchial smooth muscle contraction, and pain transmission function through the sympathetic preganglionic and postganglionic fibers in the innervation area. By blocking the reflex pathway of the spinal cord, SGB reduces the excitability of sympathetic nerves, inhibits muscle reflex and vasoconstriction, reduces the concentration of norepinephrine and prostaglandin in plasma, improves local tissue ischemia and hypoxia, takes away the inflammatory mediators that cause pain by relieving spasm, and increases local blood supply, thereby blocking the painful response. SGB can also significantly reduce the blood levels of cortisol, aldosterone, angiotensin 2,5-hydroxytryptamine, and substance P in the blood of patients with pain, enhance T-cell activity, reduce nerve inflammation, promote nerve repair, and relieve pain [11]. Previous SGB was mostly blind piercings, which require accurated positioning and careful operation. Operators are required to be proficient in neck neuromuscular anatomy and puncture techniques and be able to detect and deal with related complications in a timely manner. The requirements for the operator are higher, and the risk of independent outpatient treatment is higher. Now, the ultrasound has become conventional equipment in the field of pain; SGB under ultrasound guidance can greatly improve the accuracy and safety of the operation. According to the report by Yoo et al. [12], ultrasound-guided percutaneous SGB requires less anesthetic dose to achieve the same effect than pure percutaneous SGB, the effect is better, and adverse complications are less, and it is more suitable for regular treatment of outpatients.

As a noninvasive method, the external divergent shock wave has been used in strain diseases such as tenosynovitis, frozen shoulder, neck, shoulder, waist, and leg pain. However, the application research in neuropathic pain is still in its infancy and rarely reported at home and abroad. Shock wave therapy has a significant effect in the treatment of chronic pain, but the mechanism of its treatment of pain is still unclear. At present, it is believed that shock wave therapy mainly produces analgesia, improves microcirculation, and promotes angiogenesis through piezoelectric effect, cavitation effect, and mechanical effect. When the shock wave passes through soft tissues such as muscles, ligaments, and tendons, it produces different mechanical effects, resulting in different tension, and pressure is generated on the tissues. The tiny air bubbles in the medium expand at a high speed to loosen the tissues, reduce the adhesion of the focal lesions, promote microcirculation, and increase oxygen uptake by cells [13]. In addition, the shock wave produces superstimulation to the nerve ending tissue, causing free radical changes around the cell, reducing nonmyelinating nerves, promoting the release of substance P in painful parts, increasing cell permeability, releasing nitric oxide and changing the composition of nociceptor chemical mediators, inhibiting the transmission of pain information, and increasing the pain threshold, thereby alleviating pain [14]. At present, there are no research reports on the obvious side effects of shock waves, but combined with clinical and related reports, there may be complications such as pain, small and superficial hematomas, mild paralysis, and acupuncture sensation after shock wave treatment [15].

## 5. Conclusion

In summary, this study observes the short-term efficacy of ultrasound-guided SGB combined with ESWT in the treatment of neuralgia after herpes zoster, and the time and degree of pain relief are both high and single treatment. This method has the advantages of precise effect and simple operation; fewer complications can significantly relieve PHN, improve related sleep and mental problems, and improve the quality of life of patients. This treatment method is worthy of promotion. However, due to shortcomings such as short time, small number of cases collected, and short follow-up time, a more comprehensive treatment effect needs to be improved by further research.

## Figures and Tables

**Table 1:** Comparison of pain degree VAS after treatment in 3 groups (*X* ± *S*).

Group	Cases	Before treatment	After treatment		
			2 times	4 times	6 times
Group A	12	7.8 ± 1.3	6.8 ± 1.1^1)^	5.4 ± 1.3^1)^	3.1 ± 1.2^1)^
Group B	12	7.9 ± 0.9	6.9 ± 0.9^1)^	5.7 ± 1.3^1)^	3.3 ± 1.3^1)^
Group C	12	7.8 ± 1.0	6.0 ± 1.0^1)2)^	4.3 ± 0.8^1)2)^	1.9 ± 0.7^1)2)^

*Note.* Compared with before treatment, 1) *P* < 0.05; compared with different groups, 2) *P* < 0.05.

**Table 2:** Comparison of pain disorder index (PDI) after treatment of 3 groups (*X* ± *S*).

Group	Cases	Before treatment	After treatment		
			2 times	4 times	6 times
Group A	12	46.3 ± 12.1	37.4 ± 10.9^1)^	26.4 ± 9.7^1)^	11.7 ± 8.4^1)^
Group B	12	45.9 ± 7.2	38.7 ± 6.0^1)^	25.9 ± 9.5^1)^	12.3 ± 7.8^1)^
Group C	12	47.5 ± 7.6	33.5 ± 7.6^1)^	17.8 ± 7.7^1)2)^	4.6 ± 3.2^1)2)^

*Note.* Compared with before treatment, 1) *P* < 0.05; compared with different groups, 2) *P* < 0.05.

## Data Availability

The data used to support the findings of this study are available upon reasonable request from the corresponding author.
